The article "Prevalence, Risk Factors, and Mortality of Patients Presenting with Moderate and Severe Hyponatremia in Emergency Departments" was published in 2023. Journal: Emerg Med Int.

# Prevalence, Risk Factors, and Mortality of Patients Presenting with Moderate and Severe Hyponatremia in Emergency Departments

**DOI:** 10.1155/2023/9946578

**Published:** 2023-12-31

**Authors:** Randa Farah, Nisreen Asha, Farah Mezher, Saja Maaitah, Fedaa Abu Al-Samen, Farah Abu Abboud, Salma Ajarmeh

**Affiliations:** ^1^Nephrology Division, Internal Medicine Department, School of Medicine, The University of Jordan, Queen Rania Street, Amman 11942, Jordan; ^2^School of Medicine, The University of Jordan, Amman, Jordan; ^3^Paediatric Departments, School of Medicine, Mutah University, Karak, Jordan

## Abstract

**Background:**

Hyponatremia is among the most common electrolyte disturbances encountered in clinical practice and is associated with a high rate of morbidity and mortality. However, there are very limited data on adult cases presenting to emergency departments with hyponatremia.

**Objectives:**

This study aimed to evaluate the frequency, clinical characteristics, and outcomes in hyponatremic patients presenting to emergency departments.

**Methods:**

This retrospective study analyzed all patients older than 18 years who visited our institution's emergency department between October 2018 and October 2019 and has a serum sodium (Na) level <130 mmol/L.

**Results:**

Among 24,982 patients who visited the emergency department and had a documented serum sodium level, 284 were included. Patients' median age was 67.13 ± 14.8 years. Younger patients are less likely to develop severe hyponatremia compared to older patients (adjusted odds ratio (AOR): 0.415; 95% confidence interval (CI): 0.231–0.743; *p*=0.003). Asymptomatic hyponatremia and gastrointestinal manifestations were the most common presenting hyponatremia symptoms (33.7% and 24.2%, respectively). Proton pump inhibitor (PPI) use, angiotensin-converting enzyme inhibitor/angiotensin receptor blocker (ACE/ARB) use, and spironolactone use (OR = 2.6 and 3.9, 2.3 with a *p*=0.02, 0.03, and 0.05, respectively) were associated with increased odds of severe hyponatremia. There is no difference in the overall mortality rate within 6 months of presentation between severe and moderate hyponatremia groups (11.1% versus 16.2%, *p*=0.163).

**Conclusion:**

Moderate and severe hyponatremia are not uncommon among patients presenting to emergency departments. Moderate hyponatremia can be asymptomatic with clinical significance. Older patients, use of PPI, use of ACEi/ARBs, and spironolactone use were associated with an increased risk of severe hyponatremia compared to moderate. Further prospective analysis of a larger population is needed to confirm our findings.

## 1. Introduction

Hyponatremia is among the most common electrolyte disturbances encountered in clinical practice and is associated with a wide variety of underlying diseases and conditions [1, 2]. Hyponatremia can lead to a wide spectrum of clinical symptoms, ranging from mild to severe to even life threatening, and most common reported symptoms were nausea, vomiting, dizziness, confusion, seizures, and coma [3]. These symptoms depend on the underlying disease as well as the severity and rate of the development of hyponatremia [2]. Therefore, hyponatremia has been known as an indicator of poor prognosis in some diseases and clinical settings [4–6] and is associated with increased mortality, morbidity, and length of hospital stay [3].

Although the occurrence of hyponatremia in some clinical settings has been reported [1, 7, 8], a limited number of studies have investigated the risk factors for hyponatremia and its resultant complications, which have led to the marginalization of the role of prevention and prediction of such a high impact disturbance and its underlying conditions [9, 10].

There are some data on adult cases presenting to emergency departments with hyponatremia [10], and the risk factors and associated mortality related to hyponatremia have been studied and evaluated adequately by Correia et al. [11], but still there are very limited data from the Middle East region [12].

The aim of this study was to assess the frequency, clinical and biochemical features, clinical presentation, underlying diagnoses, and clinical outcomes of hyponatremic patients presenting to emergency departments and to determine the factors associated with the increased incidence of severe hyponatremia compared to moderate hyponatremia.

## 2. Materials and Methods

This is a retrospective study that included all patients aged >18 years who visited the Jordan University Hospital emergency department between October 2018 and October 2019. All patients with a documented serum sodium level measured as part of the KFT were included. The patients with a serum sodium (Na) level of <130 mmol/L and hyposmolar hyponatremia were included in the final analysis. We excluded patients with nonhypoosmolar hyponatremia and patients with a serum sugar level >400.

Because patients with serum glucose more than 400 mg/dl were excluded, we used 1.6 mmol/L added to the serum sodium level for every 100 mg of glycemia >100 mg/d equation to correct the sodium levels for hyperglycaemia [13].

The patients' paper-based and electronic medical records were reviewed, and the following covariates were collected from the hospital's database: baseline clinical characteristics, including patient demographics and comorbidities, such as diabetes mellitus, hypertension, chronic liver disease, pulmonary and renal diseases, active malignancies, and cardiac disease. Patients' baseline vital signs and laboratory data were also collected, and a list of home medications was reviewed.

We identified 284 patients with serum Na level <130 mmol/L who had hypoosmolar hyponatremia (measured effective serum osmolality <285 mOsm/kg), and we divided them into the following two groups according to the clinical severity of hyponatremia: group 1 comprised patients with moderate hyponatremia (serum Na level: 120–129 mmol/L) and group 2 comprised those with severe hyponatremia (serum Na level: ≤120 mmol/L). Severe hyponatremia is often defined as the plasma sodium level under 120 mmol/L and may lead to seizures, obtundation, coma, and respiratory arrest [14]. The presenting symptoms and most likely diagnoses were reviewed and analyzed. The clinical outcome was determined by the admission to the hospital versus discharge from the emergency department and mortality within 6 months after presentation.

The presenting symptoms were classified into the following categories: gastrointestinal (GI) symptoms, such as nausea, vomiting, and abdominal pain, with all surgical and medical causes having been ruled out by appropriate laboratory and imaging examinations and with the symptoms improving after correcting the Na level. Neurological symptoms, such as confusion, altered level of consciousness, seizure, and focal neurological deficit, with surgical and medical causes having been ruled out by appropriate imaging examinations and the symptoms improving after correcting the Na level; muscular symptoms, such as generalized weakness, vague muscle aches, and easy fatigability, which are not caused by other clinical diagnoses and improved after correcting hyponatremia. Moreover, patients may have two or three concomitant symptoms, indicating the presence of more than one of the abovementioned symptoms. Finally, patients may also present with asymptomatic hyponatremia, in whom no symptoms related to hyponatremia were observed and the low Na level was only found accidentally.

The clinical diagnoses were categorized as follows: respiratory diseases include lung pathologies such as acute exacerbations of chronic pulmonary diseases (e.g., chronic pulmonary disease, asthma exacerbation, lung fibrosis) and new-onset lung conditions like pneumonia that do not significantly affect hemodynamics. Acute gastroenterology: this category encompasses medical causes of gastrointestinal bleeding, decompensated liver failure, acute liver failure, and similar conditions. Acute neurological diseases: they refer to various neurological conditions, including ischemic or hemorrhagic stroke, as well as acute neurological illnesses like myasthenia gravis, Guillain–Barré syndrome, or other neuropathic diseases. Endocrinological diseases: this category involves conditions such as myxedema coma, Addisonian crisis, and cases of hypercalcemia or hypocalcemia. Acute cardiac causes: they encompass acute decompensated heart failure associated with infections or cardiac arrhythmias linked to infections, including acute myocardial infarction and others. Nephrology diagnosis: it relates to diagnoses associated with kidney diseases and disorders, such as acute kidney injury, chronic kidney disease, renal failure, and kidney stones. Infectious diagnosis: it refers to diagnoses of infectious diseases caused by pathogens such as bacteria, viruses, fungi, or parasites. Examples include bacterial pneumonia, influenza, urinary tract infection, and malaria. Malignant diagnosis: it involves diagnoses of various types of cancers, such as lung cancer, breast cancer, colorectal cancer, and leukemia. Additionally, there is a category for diagnoses that do not fit the above definitions, and it is worth noting that the initial diagnosis for presenting symptoms in this study is hyponatremia.

### 2.1. Ethics Statement

This study was conducted in accordance with the principles stipulated in the World Medical Association Declaration of Helsinki. The data were obtained from the hospital's database following the rules for release of the University Hospital. This ensured confidentiality and nondisclosure of individual identifiers. The Institutional Review Board approved the study design. The requirement for obtaining informed consent was waived for this study owing to its retrospective nature.

### 2.2. Statistical Analysis

We used SPSS version 21.0 (Chicago, USA) in our analysis. Descriptive data were summarized using means, standard deviations, frequencies, and percentages. Pearson's chi-square test of independence was used between study variables and severity of hyponatremia (univariate approach) to determine whether a statistically significant association exists between the proportions of two groups. The variables significantly associated with the severity of hyponatremia (*p* ≤ 0.05) were included in the logistic regression model to determine the odds ratio (OR) of clinically significant data and to explore the possible associated factors and outcomes with the severity of hyponatremia. We adopted a *p* value of 0.05 as the significant threshold.

## 3. Results

### 3.1. Patient Characteristics

Among 24,982 patients aged >18 years who visited the emergency department between October 2018 and October 2019 and had documented serum sodium level measured as part of the KFT, 874 (3.5%) patients had hyponatremia (Na *l* < 135) and hypotonic hyponatremia.

We found that 284 (1.136%) patients had moderate-to-severe hyponatremia, as indicated by a serum Na level of <130 mmol/L (185 patients had their serum sodium (121–129 mmol/L) and 99 patients ≤120 mmol/L) (Figure 1).

The patients' baseline characteristics were recorded according to the severity of hyponatremia (Table 1). The median age of our study population was 67.13 ± 14.8 years. There were 115(40.5%) men and 169 (59.5%) women. There was a significant difference in age between the moderate and severe hyponatremia groups, as older patients were more likely to have severe hyponatremia (≤120 mmol/L; *p*=0.001). No significant differences were found in sex, systolic blood pressure, diastolic blood pressure, heart rate, and serum potassium (K), and serum creatinine, serum hemoglobin, and serum albumin levels between groups 1 and 2 (Table 1). Furthermore, there is no significant association between the severity of hyponatremia and other comorbidities (Table 1).

Regarding the patients' home medications, we found a statistically significant difference between the moderate and severe hyponatremia groups. The patients who were using angiotensin-converting enzyme inhibitors/angiotensin receptor blockers (ACEi/ARBs), beta blockers, spironolactone, gabapentin, and proton pump inhibitors (PPI) were at a higher risk of developing severe hyponatremia than those not taking these medications (*p*=0.03, 0.008, 0.01, 0.009, and 0.008, respectively). In addition, we found that tricyclic antidepressants were associated with moderate hyponatremia (*p*=0.05).

### 3.2. Symptoms of Hyponatremia and Clinical Diagnoses

Among the patients, the most common presentation of hyponatremia was asymptomatic hyponatremia, which occurred in 96 (33.7%) patients, and the second most common was GI symptoms, which occurred in 69 (24.2%) patients (Table 2). A significant correlation was observed between the severity of hyponatremia and clinical presentation, as almost 40% of patients in group 1 were asymptomatic, while 24% of patients in group 2 presented with two concomitant symptoms (*p*=0.04) (Table 2).

The most common diagnosis at the emergency room that were related to the presentation of a low serum Na level was hyponatremia (29.9%), followed by cardiac and pulmonary diseases (14.7% and 14.4%, respectively) (Table 2). There was no significant association found between the severity of hyponatremia and clinical diagnosis (*p*=0.87).

### 3.3. General Outcome

Regarding the patients' outcomes, which included admission to the hospital and mortality, 88.1% and 99% of the patients in groups 1 and 2, respectively, were admitted to the hospital, with the difference being statistically significant (*p*=0.001). The overall mortality rate within 6 months of presentation was 11.1% and 16.2% for groups 1 and 2, respectively, with the difference being nonsignificant between the two groups (*p*=0.16) (Table 3). The patients who were discharged were managed at the emergency department for their hyponatremia and sent home after correction.

### 3.4. Logistic Regression

The results were further adjusted using a logistic regression to determine the effects of age groups, chronic liver disease, clinical presentation, use of beta blockers, ACEi/ARBs, other diuretics (spironolactone), PPIs, and gabapentin, and clinical outcomes, which are the study variables that were clinically significant in the chi-square test (*p* < 0.01). The logistic regression model was found to be statistically significant (*χ*^2^ (9) = 70.5, *p* < 0.001). The model explained 30.8% (Nagelkerke *R*^2^) of the variance in severe hyponatremia (Na level ≤120 mmol/L) and correctly classified 93.4% of the cases. Of the eight predictor variables, five predictors, including age, clinical presentation (two concomitant symptoms), use of ACEi/ARBs, use of PPIs, and clinical outcome, were statistically significant. Younger patients (age <65 years) had a lower risk of developing severe hyponatremia than older patients (age >65 years) (adjusted OR (AOR): 0.42; 95% confidence interval (CI): 0.23–0.74; *p*=0.003). Patients with severe hyponatremia were more likely to have two concomitant symptoms compared to patients with moderate hyponatremia, with asymptomatic hyponatremia being the reference asymptomatic (AOR: 3.69; 95% CI: 1.61–8.48; *p*=0.002). In addition, patients with severe hyponatremia were more likely to be admitted to the hospital compared to patients with moderate hyponatremia (AOR: 11.25; 95% CI: 1.10–114.78; *p*=0.04). Patients who are not taking ACEi, PPI, and spironolactone had a lower risk of developing severe hyponatremia than who are taking their medications (AOR: 0.38, 0.26, and 0.43, respectively), with the difference being statistically significant (*p*=0.02, 0.03, and 0.05, respectively; Table 3).

## 4. Discussion

In this study, the incidence of hyponatremia, as indicated by a serum sodium level of <135 mmol/L, was approximately 3.5% and that is comparable to the overall incidence of hyponatremia reported among previous studies, which ranged from 3% to 7% depending on the definitions of the disturbance and the population surveyed [15, 16]. In addition to that, we found that the incidence of moderate-to-severe hyponatremia, defined as the serum sodium level of <130 mEq/L, was approximately 1.14% and it is comparable to what was reported by Olsson et al. [16].

In this study, 34.9% of patients had severe hyponatremia (≤120 mmol/L), and 65.1% had moderate hyponatremia (120–135). Severe hyponatremia is often defined as the serum Na level ≤120 mmol/L and associated with more severe symptoms and may lead to seizures, obtundation, coma, and respiratory arrest [14]. In a retrospective cross‐sectional study, the risk of seizures in hyponatremia patients were higher at serum Na levels <110 mmol/L with an odds ratio of 18.06 (95% CI: 1.96–166.86) as compared to the plasma sodium Na level of 120–124 mmol/L [17].

The patients in the present study were an older population, with a mean age of 67.1 ± 14.8 years. This is consistent with the findings of a previous study reporting that patients with an older age are more likely to have severe hyponatremia [18]. In this study, patients aged >65 years had 2.65 times increased risk of developing severe hyponatremia compared to the risk of developing moderate hyponatremia. Several studies have reported that elderly people are considered at a high risk for developing hyponatremia, and advanced age is considered a strong independent risk factor for hyponatremia [19]. However, our study population was older than those of several published studies, which reported a mean age of approximately 55 years [18].

Twenty-three percent of patients with Na ≤120 mmol/L had asymptomatic hyponatremia, whereas 39% of those who had hyponatremia of 120–130 mmol/L were asymptomatic, and their hyponatremia was only accidentally found. This means that hyponatremia can be serious and asymptomatic, and those with severe hyponatremia were more likely to have more than one symptom of hyponatremia. In addition, the most common presenting symptoms among the study population were GI manifestations, whereas, in the severe hyponatremia (≤120 mmol/L) and moderate hyponatremia (120–130 mmol/L) groups, the most common presentations were the two concomitant symptoms and asymptomatic presentation, respectively.

Our findings were different from those reported by Braun and his colleagues who demonstrated that patients with hyponatremia mostly present with mental status changes (40%), nausea and vomiting (30%), and generalized weakness (30%) [20]. On the other hand, other reports showed that patients with profound hyponatremia usually show nonspecific neurological symptoms and may undergo neuroimaging examinations unnecessarily. Bokemeyer et al. found that, among the 52,918 emergency admissions and 261 patients with profound hyponatremia, 140 (54%) had neurological symptoms [21]. Unspecific weakness and confusion were the most prevalent symptoms (59%). Focal neurological signs were present in 31% of cases, and neuroimaging examinations were performed on 68% (95/140) of symptomatic patients.

Our study did not find the increased risk of moderate or severe hyponatremia in patients who are receiving thiazide diuretics and that can be related to small size sample and small number of patients who are taking thiazide or patients stopped it earlier because of mild hyponatremia.

Our study showed that the use of ACEi/ARBs increases the risk of severe hyponatremia by 3.9 times compared to the risk of moderate hyponatremia (*p*=0.027), which is in line with the finding reported by Bhuvaneshwari et al., who concluded that hyponatremia was induced in nearly 50% of patients taking ACEi and ARBs, although the incidence of hyponatremia between patients receiving ACEi and those receiving ARBs were not statistically different [21]. In addition, they explained that the mechanism of ACEi- and ARB-induced hyponatremia has not been confirmed, but ACEi therapy increased the circulating angiotensin I that enters the brain and is converted into angiotensin II, which may stimulate thirst and release of antidiuretic hormone from the hypothalamus, eventually leading to hyponatremia [22, 23]. A previous report also indicated that there is a blockade of aldosterone-induced renal tubular Na reabsorption and K secretion, which might lead to the lowering of serum Na levels [24].

We found that 10.5% of patients were taking other diuretics (spironolactone), and the proportion of patients with severe and moderate hyponatremia was 56% and 7%, respectively, with the difference being statistically significant. Therefore, patients taking spironolactone are more likely to have severe hyponatremia. This is supported by a previous study that described spironolactone-related hyponatremia in the following two contexts: the first is the treatment of severe heart failure and liver failure, and the second is resistant hypertension unrelated to hyperaldosteronism. The study further demonstrated that spironolactone is frequently used in heart failure and liver cirrhosis, where dilutional hyponatremia is indicative of a decompensated underlying disease. In addition, spironolactone is commonly used with loop diuretics in patients with heart failure, and the hyponatremia in this case was considered to be due to the excessive natriuretic response to spironolactone [25].

Tricyclic antidepressants were found to be protective against hyponatremia, as patients who took tricyclic antidepressants were found less likely to be at a high risk for severe hyponatremia. However, the relationship between the use of tricyclic antidepressants and hospitalization due to hyponatremia was small to moderate. In contrast, there was no evidence showing that continuing treatment with antidepressants increases the risk of hospitalization due to hyponatremia [26].

In the present study, PPI use increased the risk of severe hyponatremia by 2.6 times, compared to the risk of moderate hyponatremia. Small observational studies and case reports have indicated that PPIs may cause hyponatremia [27]. Whether there is a difference in the risk of severe hyponatremia among the individual PPI remains unknown. Given that PPIs are one of the most commonly prescribed groups of drugs, even a rare adverse reaction may have large implications. A study that investigated the association between PPIs, with the exception of lansoprazole, and hospitalization due to hyponatremia suggested an association between any newly initiated PPI treatment and hospitalization due to hyponatremia. Ongoing PPI use was not associated with an increased risk of hyponatremia [28]. In addition, another study on hyponatremia involving elderly (age >65 years) assessed the risk of hyponatremia between patients exposed to PPIs for at least 1 year and controls not exposed to the PPIs. The study showed that the risk of moderate hyponatremia is increased by chronic use of PPIs in the elderly population [29].

We observed that patients taking gabapentin were more likely to have severe hyponatremia, but the difference was not statically significant in the logistic regression analysis. Wilton and colleagues conducted a postmarketing observational cohort study of gabapentin as an add-on therapy for 3,100 patients and showed that, at 6 months after its prescription, two patients developed hyponatremia; however, there was little information about the cases [28]. In one of these cases, the patient continued with gabapentin treatment, and the Na levels remained low. In the second case, the patient's Na levels returned to normal values after gabapentin discontinuation [30]. Several reviews of hyponatremia in the elderly and its challenges and solutions found that carbamazepine and oxcarbazepine are the most common antiepileptic drugs that are associated with hyponatremia. Recently, other antiepileptic drugs, such as gabapentin, have also been reported to induce hyponatremia [19].

In the severe hyponatremia group, most of our patients were admitted to the hospital. This is the appropriate management of severe hyponatremia, and this amount of admission is a burden on the hospital; thus, we need to carefully examine patients with severe hyponatremia and consider it a serious comorbidity. Callahan and colleagues conducted a cohort study of hospitalized patients (age ≥18 years) with hyponatremia at admission and found that patients with mild-to-moderate and moderate-to-severe hyponatremia had significantly longer and more costly hospitalizations than patients with normonatremia [31]. Another study reported that, on admission, 25.2% of patients had moderate hyponatremia (126–129 mmol/L) and 3.6% had severe hyponatremia (<126 mmol/L) [32].

The mortality rate within 6 months of admission in our sample was 14.4%. Winzeler and his colleagues proposed, in a follow-up study of patients with profound hyponatremia (≤125 mmol/L) admitted to the emergency department, that hyponatremia is associated with increased one-year mortality, recurrence, and rehospitalization rates [33]. The study showed that, during the follow-up period, 20.6% of patients died. In addition, Hao and colleagues conducted a cohort study involving 154,378 adults who were hospitalized between 2008 and 2012 at a teaching hospital in Beijing and found that the mortality risk increased with increasing severity of hyponatremia in all diagnostic groups. The overall in-hospital mortality rate was 6.15% in patients with hyponatremia, whereas that of patients without hyponatremia was 0.48% [6]. Moreover, Zieschang and colleagues concluded that the in-hospital mortality was five times higher in the hyponatremia group than in the control group. Castello et al. and his group found moderate-to-severe hyponatremia at ED presentation independently predict mortality in septic patients, and this can help in early risk stratification and suggest more aggressive therapeutic strategies [34]. After 6 months, the outcomes of the hyponatremia group were worse (mortality: 32% versus 23%, *p*=0.080; mortality or institutionalization: 46% versus 35%, *p*=0.067) [35].

### 4.1. Limitations

This study has a few limitations. First, the present work was a retrospective and single-center study with a limited number of patients. Second, all clinical data were obtained from the emergency room evaluation sheets, which can have missing data related to the final diagnosis. Third, we were unable to assess the patients' volume status and could not determine the type of hyponatremia. We also do not have data on urine osmolality or spot urine Na for all patients. We could not include some neurological symptoms as memory loss and mild cognitive dysfunction, as those are not usually clinical symptoms patients present in the emergency room. Finally, we did not assess the treatment plan for these patients or follow up the cause of their deaths.

## 5. Conclusion

Moderate and severe hyponatremia is not uncommon among patients presenting to emergency departments and associated with a high mortality rate. Patients with severe hyponatremia presented with more than one symptom, mostly two concomitant symptoms. Moderate hyponatremia can be asymptomatic with clinical significance. Severe hyponatremia is seen in older patients and in those taking ACEi/ARBs, PPIs, and spironolactone. Physicians should be aware of the severity of hyponatremia, its various clinical presentations, and clinical outcomes. Further prospective analysis of a larger population is needed to confirm our findings.

## Figures and Tables

**Figure 1:** Flow chart of patients included and excluded in the study.

**Table 1:** Baseline characteristics of the 257 patients grouped according to the severity of hyponatremia (univariate associations).

	Group 1: Na = 121–130 mmol/L *n* = 185 (65.1%)	Group 2: Na ≤ 120 mmol/L *n* = 99 (34.9%)	Total	Chi-square
*Demographics*:				
Age				
>65	98 (53.0%)	72 (72.7%)	170 (59.9%)	0.001^*∗*^
<65	87 (47.0%)	27 (27.3%)	114 (40.1%)	
Mean age (year) ± SD	69.9 ± 14.16	65.65 ± 15	67.13 ± 14.8	
Gender				
Male	80 (43.2%)	35 (35.4%)	115 (40.5%)	0.12
Female	105 (56.8%)	64 (64.9%)	169 (59.5%)	

*Blood pressure: (Mean)*				
Systolic blood pressure	133 ± 29.8	134.04 ± 31.4	133.7 ± 30.83	0.77
Diastolic blood pressure	72 ± 18.44	74 ± 17.75	73 ± 19	0.87
Heart rate	78.5 ± 18.32	83.7 ± 16.85	81.9 ± 17.52	0.27

*Biochemical values: (Mean)*				
Potassium (mmol/L)	4.43 ± 0.96	4.7 ± 3.0	4.62 ± 2.52	0.4
Serum albumin (g/L)	31.6 ± 13.8	28.5 ± 15.9	29.6 ± 15.2	0.2
Serum hemoglobin level (g/L)	118.2 ± 30.0	118.9 ± 36.0	118.6 ± 34.0	0.9
Serum creatinine (mmol/L)	128.0 ± 141.0	123.1 ± 164.7	128.0 ± 141.0	0.5
Serum glucose (mmol/L)	10.4 ± 6.0	10.0 ± 5.6	10.2 ± 5.7	0.9

*Comorbidities*:				
Diabetes	114 (61.6%)	69 (69.7%)	183 (64%)	0.18
Hypertension	140 (75.7%)	82 (82.8%)	222 (77.9%)	0.16
Cardiac disease	65 (35.1%)	44 (44.4%)	109 (38.2%)	0.12
Neurological disease	26 (14.1%)	12 (12.1%)	38 (13.3%)	0.65
Chronic pulmonary disease	25 (13.5%)	13 (13.1%)	38 (13.3%)	0.93
Chronic liver disease	8 (4.3%)	10 (10.1%)	18 (6.3%)	0.06
Malignancy	21 (11.4%)	9 (9.1%)	30 (10.5%)	0.56
Chronic kidney disease	37 (20.0%)	22 (22.2%)	59 (20.7%)	0.66
Seizure disorder	9 (4.9%)	2 (2%)	11 (3.9%)	0.24

*Medications*:				
ACEi/ARBs	56 (30.3%)	43 (43.4%)	99 (34%)	0.03^*∗*^
Beta blockers	74 (40%)	56 (56.6%)	130 (45.6%)	0.008^*∗*^
Thiazide diuretics	36 (19.5%)	15 (15.2%)	51 (17.9%)	0.34
Loop diuretics	82 (44.3%)	52 (52.5%)	134 (47.0%)	0.25
Spironolactone	13 (7%)	17 (56.7%)	30 (10.5%)	0.01^*∗*^
Tricyclic antidepressants	7 (3.8%)	0 (0%)	7 (2.5%)	0.05^*∗*^
Selective serotonin reuptake inhibitors	7 (3.8%)	2 (2.1%)	9 (3.2%)	0.40
Carbamazepine	17 (9.2%)	9 (9.1%)	26 (9.1%)	0.98
Gabapentin	12 (6.5%)	16 (16.2%)	28 (9.8%)	0.009^*∗*^
Proton pump inhibitors	93 (50.3%)	66 (66.7%)	159 (55.8%)	0.008^*∗*^
NSAIDs	9 (4.9%)	5 (5.1%)	14 (4.9%)	0.95

**Table 2:** Hyponatremia symptoms and clinical diagnosis.

	Group 1: Na = 120–130 mmol/L	Group 2: Na ≤ 120 mmol/L	Total (%)	Chi-square
*Presenting symptoms: (Count, %)*				
Gastrointestinal symptoms	44 (23.8%)	25 (25.3%)	69 (24.2%)	0.04^*∗*^
Neurological symptoms	25 (13.5%)	11 (11.1%)	36 (12.6%)	
Muscular symptoms	12 (6.5%)	12 (12.1%)	24 (8.4%)	
Two concomitant symptoms	26 (14.1%)	24 (24.2%)	50 (17.5%)	
Three concomitant symptoms	5 (2.7%)	4 (4.0%)	9 (3.2%)	
Asymptomatic	73 (39.5%)	23 (23.2%)	96 (33.7%)	

*Clinical diagnosis: (Count, %)*				
Respiratory diagnosis	26 (14.1%)	15 (15.2%)	41 (14.4%)	0.87
Endocrinological diagnosis	19 (10.3%)	6 (6.1%)	25 (8.8%)	
Cardiac diagnosis	28 (15.1%)	14 (14.1%)	42 (14.7%)	
Malignant diagnosis	2 (1.1%)	2 (2.0%)	4 (1.4%)	
Neurological diagnosis	6 (3.2%)	1 (1%)	7 (2.5%)	
Nephrology diagnosis	21 (11.4%)	14 (14.1%)	35 (12.3%)	
Infectious diagnosis	12 (6.5%)	8 (8.1%)	20 (7.0%)	
Other diagnosis	17 (9.2%)	8 (8.1%)	25 (8.8%)	
Hyponatremia	54 (29.2%)	31 (31.3%)	85 (29.9%)	

*Hospital outcome: (Count, %)*				
Admitted to the hospital	163 (88.1%)	91 (99.0%)	0.001^*∗*^	
Discharged home	22 (11.9%)	1 (1.0%)		

*Mortality: within 6 months*				
Overall mortality 41 (14.4%)	11 (11.1%)	30 (16.2%)	0.16	

**Table 3:** Logistic regression analysis of the study variables for severe hyponatremia.

Variables	Odds ratio	95% CI lower	Upper	*p* value
Age group				0.003^*∗*^
<65	0.42	0.23	0.74	
>65	1	Reference		
Clinical presentation				
Gastrointestinal symptoms	1.97	0.94	4.14	0.07
Neurological symptoms	1.42	0.57	3.57	0.46
Muscular symptoms	2.05	0.74	5.69	0.17
Two concomitant symptoms	3.69	1.61	8.48	0.002^*∗*^
Three concomitant symptoms	2.23	0.49	10.05	0.3
Asymptomatic	1	Reference		
B blocker use				0.14
No	0.53	0.23	1.24	
Yes	1	Reference		
Spironolactone use				0.05^*∗*^
No	0.43	0.18	0.95	
Yes	1	Reference		
Proton pump inhibitors				0.02^*∗*^
No	0.38	0.17	0.88	
Yes	1	Reference		
Gabapentin use				0.83
No	0.1.157	0.37	4.22	
Yes	1	Reference		
ACEi/ARBs' use				0.03^*∗*^
No	0.26	0.075	0.87	
Yes	1	Reference		
Admission outcome				0.04^*∗*^
Admission	11.25	1.10	114.78	
Discharge home	1	Reference		

## Data Availability

The datasets used and/or analyzed during the current study are available from the corresponding author on request.

## Additional Points

*Article Summary*. Why is this topic important? Hyponatremia is one of the most common electrolyte disturbances and is associated with a high rate of morbidity and mortality. There are very limited data on adult cases presenting to emergency departments with hyponatremia and clinical presentation with clinical outcomes. What does this study attempt to show? The frequency of hyponatremia in our population and the clinical presentation and outcomes in hyponatremic patients presenting to emergency departments. What are the key findings? (i) Moderate and severe hyponatremia can be asymptomatic and accidentally found and associated with significant adverse clinical outcomes. Our findings were different from many observational studies which demonstrate that patients with hyponatremia mostly present with mental status changes and other serious symptoms. (ii) Whether there is a difference in the risk of severe hyponatremia among the individual uses of PPI remains unknown, and our study showed that the use of PPI increased the risk of severe hyponatremia. (iii) This study provides more information about moderate and severe hyponatremia in regard with frequency, clinical presentation, risk factors, and mortality in emergency department patients. How is patient care impacted? Emergency physicians should be aware of the severity of hyponatremia, its various clinical presentations, and clinical outcomes. That will help in proactive treatment of hyponatremia and further evaluation.
